The article "Identification of genuine primary pulmonary NK cell lymphoma via clinicopathologic observation and clonality assay" was published in 2013. Journal: Diagn Pathol.

# Identification of genuine primary pulmonary NK cell lymphoma via clinicopathologic observation and clonality assay

**DOI:** 10.1186/1746-1596-8-140

**Published:** 2013-08-19

**Authors:** Li Gong, Long-Xiao Wei, Gao-Sheng Huang, Wen-Dong Zhang, Lu Wang, Shao-Jun Zhu, Xiu-Juan Han, Li Yao, Miao Lan, Yan-Hong Li, Wei Zhang

**Affiliations:** 1 The Helmholtz Sino-German Laboratory for Cancer Research, Department of Pathology, Tangdu Hospital, the Fourth Military Medical University, Shaanxi Xi’an 710038, China; 2 Department of Nuclear Medicine, Tangdu Hospital, the Fourth Military Medical University, Shaanxi Xi’an 710038, China

**Keywords:** Extranodal NK/T cell lymphoma, Lung, Immunophenotype, TCR gene rearrangement, Clonality

## Abstract

**Abstract:**

Extranodal natural killer (NK)/T-cell lymphoma, nasal type, is an uncommon lymphoma associated with the Epstein-Barr virus (EBV). It most commonly involves the nasal cavity and upper respiratory tract. Primary pulmonary NK/T cell lymphoma is extremely rare. If a patient with a NK or T-cell tumor has an unusual reaction to treatment or an unusual prognosis, it is wise to differentiate NK from T-cell tumors. The clinicopathologic characteristics, immunophenotype, EBV in situ hybridization, and T cell receptor (TCR) gene rearrangement of primary pulmonary NK cell lymphoma from a 73-year-old Chinese woman were investigated and the clonal status was determined using female X-chromosomal inactivation mosaicism and polymorphisms at the phosphoglycerate kinase (PGK) gene. The lesion showed the typical histopathologic characteristics and immunohistochemical features of NK/T cell lymphoma. However, the sample was negative for TCR gene rearrangement. A clonality assay demonstrated that the lesion was monoclonal. It is concluded that this is the first recorded case of genuine primary pulmonary NK cell lymphoma. The purpose of the present work is to recommend that pathologists carefully investigate the whole lesion to reduce the likelihood that primary pulmonary NK cell lymphoma will be misdiagnosed as an infectious lesion. In addition, TCR gene rearrangement and clonal analysis, which is based on female X-chromosomal inactivation mosaicism and polymorphisms at PGK and androgen receptor (AR) loci, were found to play important roles in differentiating NK cell lymphoma from T cell lymphoma.

**Virtual slides:**

The virtual slide(s) for this article can be found here: http://www.diagnosticpathology.diagnomx.eu/vs/5205300349457729

## Introduction

Extranodal NK/T cell lymphoma, nasal type, is a rare form of lymphoma. It often involves the nasal cavity and usually presents as destructive lesions within the midline facial structures. For this reason, it used to be called “lethal midline granuloma”. It has also been reported that, in addition to the nasal cavity, NK/T cell lymphoma can arise in the skin, gastrointestinal tract, testes, brain, salivary glands, pancreas, soft tissues, adrenal glands, and bone marrow [1-3]. Although this illness can occur at any age, it appears more often in people in their 50s and affects more men than women [4,5]. Primary pulmonary NK/T cell lymphoma is extremely rare. To the best of our knowledge, only four cases have been reported in the English-language journals [6-8]. Histopathologically, these lesions usually show extensive coagulative necrosis with atypical lymphocyte infiltration. They are often misdiagnosed as infarction or chronic inflammation if large numbers of specimens are not carefully evaluated by pathologists. No case of genuine primary pulmonary NK cell lymphoma has yet been reported in English. In the present study, a case of primary pulmonary NK cell lymphoma from a 73-year-old Chinese female patient is reported and its clinicopathological characteristics, immunophenotype, EBV in situ hybridization, T cell receptor (TCR) gene rearrangement, and clonality are described.

The article "Identification of genuine primary pulmonary NK cell lymphoma via clinicopathologic observation and clonality assay" was published in 2013. Journal: Diagn Pathol.

## Materials and methods

### Sample

A 73-year-old female was referred to our hospital due to a 2-month history of fever up to 38.5°C. At first, the patient thought that she had a cold and took oral antibiotics for 2 weeks. However, the fever did not resolve, so she was subsequently admitted to a local hospital for further study. A chest X-ray and computed tomography (CT) showed that her right upper lung was atelectatic, and tuberculosis was considered. The patient was then treated with antituberculosis drugs for 2 weeks, but her condition did not improve, so she came to Tangdu hospital for further surgical management. Upon admission, her blood count was normal, her human immunodeficiency virus (HIV) test was negative, and she had normal lactic acid dehydrogenase (LDH) levels of 130 U/L. In addition, her plasma Epstein-Barr virus (EBV) DNA levels were 900 copies/ml. A repeat chest X-ray and CT revealed a space-occupying lesion in the upper lobe of right lung (Figure 1), which indicated central lung cancer with atelectasis of the right upper lung. Simultaneously, a nodule was found in the left upper lung. Based on these results and at the request of her family, resection of her right upper lung was performed. Written informed consent was obtained from the patient and the protocol was approved by the Institutional Ethics Committee of the Fourth Military Medical University based on the Helsinki Declaration. During the operation, a mass with an ill-defined boundary was found in lung parenchyma neighboring to the hilum of lung. The mass was dark red and medium in texture. A frozen section examination was performed in order to determine the nature of the lesion. Macroscopically, the lesion showed extensive coagulative necrosis and no evidence of malignancy.

The article "Identification of genuine primary pulmonary NK cell lymphoma via clinicopathologic observation and clonality assay" was published in 2013. Journal: Diagn Pathol.

**Figure 1:** **A chest X-ray and CT revealed a space-occupying lesion in the upper lobe of right lung.** A chest X-ray and CT revealed a space-occupying lesion in the upper lobe of right lung, which indicated central lung cancer with atelectasis of the right upper lung.

## Methods

### Immunohistochemistry and in situ hybridization

Immunohistochemical staining was performed using a streptavidin-labeled peroxidase (S-P) KIT (KIT9730,XXX) according to the manufacturer’s instructions. The primary antibodies used in this study included mouse anti-human monoclonal antibodies against leukocyte common antigen (LCA), CD2, CD3, CD3ϵ, CD20, CD45RO, CD30, CD15, CD56, CD68, CD99, BCL-2, BCL-6, latent membrane protein (LMP) 1, epithelial membrane antigen (EMA), and pan-cytokeratin (CK), CK18, rabbit anti-human polyclonal antibodies against thyroid transcription factor 1 (TTF-1), Ki-67, surfactant protein B (SP-B), S-100 protein, and smooth muscle actin (SMA), and an anti-pig monoclonal antibody against vimentin. All reagents were supplied by Maixin Biotechnology Corp. Ltd. (Fuzhou, China) but LMP 1 was from Abcam (Cambridge, UK). EBV was detected by in situ hybridization for EBER1 according to manufacturer’s instructions.

### Laser microdissection and DNA extraction

Eight 10 μm tissue sections (1.5×1.5 cm^2^) were cut from representing paraffin blocks and placed on a UV-absorbing membrane. They were subjected to laser microdissection using an LMD6000 (Leica Microsystems Ltd, Wetzlar, Germany). After hematoxylin and eosin (H&E) staining, the slides were mounted on a microstat, and the lymphoid cells were then dissected using a UV laser in motorized optical beam scanning mode. The dissectate (with the attached specimen) was dropped by gravity into the cap of a 0.5 mL microcentrifuge tube that was filled with 40 μL lysate buffer and 10 μL proteinase K. For each dissected lesion, a similar volume of surrounding normal lung tissue was isolated and analyzed as a control. The microcentrifuge tubes were then placed in a water bath (48°C) to digest the tissues. After digestion for 12 to 20 h, genomic DNA was extracted using the DNeasy Blood & Tissue Kit (Qiagen, Germany), examined using 2% agarose gel electrophoresis, and stored at -20°C.

### Polymerase chain reaction (PCR) analysis of TCR

PCR for assessment of T cell receptor gene rearrangement was performed as described by InVivoScribe Technologies, San Diego, CA (http://www.invivoscribe.com) and Bruggemann et al*.*[9]. The reaction conditions were developed for a final volume of 50 μL, consisting of 100 ng DNA, 200 μM dNTP, 10 pmol of each primer irrespective of total numbers of primers in each multiplex PCR tube, 1.5 mM MgCl_2_, and 1 U of Taq enzyme. Amplification was performed using a PT-200 thermal cycler (MJ Research, Inc., MA, U. S.) for 35 cycles (denaturation at 95°C for 30 s, annealing at 60°C for 40 s, and extension at 72°C for 30 s). The products of TCR gene rearrangement were visualized using polyacrylamide gel electrophoresis.

The article "Identification of genuine primary pulmonary NK cell lymphoma via clinicopathologic observation and clonality assay" was published in 2013. Journal: Diagn Pathol.

### PCR amplification for clonal assay

Nested PCR was used to detect single nucleotide polymorphism (SNP) sites in the PGK, as described previously [10]. Ten-microliter aliquots of genomic DNA extracted from lesion and non-lesion tissue samples were digested with 5 U of *Hpa* II (Promega, WI, U.S.) at 37°C for 3 h in a 20 μL reaction containing 0.2 μL bovine serum albumin (BSA; 10 g/L) and 2 μL 10× reaction buffer. Then 5 μL aliquots of digested DNA samples were subjected to nested PCR. The 50 μL reaction mixture consisted of 4 μL of 10 mM dNTPs (Gibco BRL, Life Technologies, Inc., MD, U.S.), primers PGK1A and PGK1B (0.4 pmol each), 5 μL of 10× buffer, 1.5 μL of 50 mM MgCl_2_, and 2.5 U of Taq DNA polymerase (Gibco BRL, MD, U.S.). Amplification was performed using a PT-200 thermal cycler (MJ Research, Inc., MA, U. S.) for 25 cycles (denaturation at 94°C for 40 s, annealing at 56°C for 50 s, and extension at 72°C for 1 min). PCR products from the first round (5 μL) were used as a template for the second PCR reaction, which was carried out with PGK2A and PGK2B primers using the same amplification protocol. The PCR products were digested with 5 U of *Bst* XI at 48°C for 8 to 10 h in a 20 μL reaction containing 0.2 μL of BSA (10 g/L) and 2 μL of 10× reaction buffer. The digested products were visualized using 2% agarose gel electrophoresis.

### Analysis and assessment of PCR products for clonality assay

PCR gel images were recorded, and the PCR band intensities for both alleles were quantitated using an image-analyzing system (LabWorks 3.0, UVP, Cambridge, U.K.). Loss of X chromosome inactivation mosaicism was defined as a reduction in the intensity of fluorescence (≥ 50%) for either band relative to that of PCR products that did not undergo digestion. A corrected ratio (CR) was calculated as the ratio of the intensity of the upper band to that of the lower band before digestion divided by the ratio of that of the upper band intensity to that of the lower band intensity after digestion. In the present study, a CR value ≥2 was used to define loss of X chromosome inactivation mosaicism.

The article "Identification of genuine primary pulmonary NK cell lymphoma via clinicopathologic observation and clonality assay" was published in 2013. Journal: Diagn Pathol.

## Results

### Pathological observation

Grossly, the mass measured 5 cm × 4 cm × 4 cm, and the cut surface was dark red. Microscopically, the lesion showed extensive coagulative necrosis. However, alveolar septa existed in some areas in which some medium-sized atypical lymphoid cells with round to slightly irregular nuclei were disseminated. Some tumor cells were angiocentric and angiodestructive. Mitotic figures were easily found (Figure 2). Immunohistochemically, the tumor cells were strong positive for CD56, CD3ϵ, TIA1 (Figure 3), and weak positive for LMP1, and negative for CD5, CD8, CD20, CD79a, CgA, Syn, SCLC, CK, EMA, CD99, CD10, TdT, PAX-5, and BCL-6. EBV in situ hybridization revealed the tumor cells to be positive (Figure 3D).

**Figure 2:** **The histopathological characteristics of the lesion.** The lesion showed extensive coagulative necrosis. However, alveolar septum existed in some areas, in which some medium-sized atypical lymphoid cells with round to slightly irregular nuclei disseminated. Moreover, some tumor cells were angiocentric and angiodestructive. Mitotic figures were easily found. (Figure 2A, 200×; Figure 2B, 200×; Figure 2C, 400×; Figure 2D, 200×).

**Figure 3:** **The immunohistochemical features and EBV in situ hybridization of the lesion.** Immunohistochemically, the tumor cells were positive for CD56 (Figure 3A, 200×), CD3ϵ (Figure 3B, 200×), and TIA-1 (Figure 3C, 200×); the tumor cells was positive for EBV in situ hybridization (Figure 3D, 200×).

### TCR gene rearrangement-comment

Lanes 1 and 2 showed the TCRGA and TCRGB reaction tubes, respectively. Lane 3 showed the TCRD reaction tube. Lanes 5, 6, and 7 showed the TCRBA, TCRBB, and TCRBC reaction tubes. The results, which included a positive control, showed no band and no evidence of a clonal gene rearrangement (Figure 4).

**Figure 4:** **The results of TCR gene rearrangement.** Lanes 1 and 2 indicated TCRGA and TCRGB reaction tube, respectively; lane 3 indicated TCRD reaction tube; lanes 5,6, and 7 indicated TCRBA, TCRBB, and TCRBC reaction tube, respectively; lane 9 indicated positive control; lane 10 indicated negative control.

### Determination of clonality

In the clonality assay, DNA samples analyzed without *Hpa* II digestion showed two bands of equal intensity. When DNA samples of the lesions were digested with *Hpa* II, the down bands disappeared (Figure 5). These results indicated that the lesion was monoclonal and neoplastic. However, the intensities of the two bands were equal to those of the surrounding normal lung tissues treated with and without *Hpa* II.

**Figure 5:** **The results of clonality based on X-chromosomal inactivation mosaicism and polymorphisms of PGK gene.** The clonality assay demonstrated that DNA samples analyzed without *Hpa* II digestion showed two bands of equal intensity. When DNA samples of the lesions were digested with *Hpa* II, the down bands disappeared.

The article "Identification of genuine primary pulmonary NK cell lymphoma via clinicopathologic observation and clonality assay" was published in 2013. Journal: Diagn Pathol.

### Diagnosis and outcome

Based on the histopathological characteristics outlined above and on immunohistochemical features and the results of TCR and PGK gene polymorphism analysis, the patient was finally diagnosed with primary pulmonary extranodal NK cell lymphoma. However, her family did not believe this diagnosis and refused further treatment. The patient had a persistent fever up to 39.4°C after surgical excision. Most antibiotics were ineffective against the fever, and only oral indomethacin anti-fever tablets showed any results. The condition did not improve until 15 days after the operation. The patient died one month after leaving the hospital.

## Discussion

Primary pulmonary lymphoma (PPL) is defined as an extranodal lymphoma that only arises from the lung parenchyma or bronchus [11]. PPL is rare, accounting for 3–4% of all extranodal lymphomas [12]. Most cases reported in the lungs are B-cell non-Hodgkin’s lymphoma (NHL) [13]. Non-B cell lymphomas, including T-cell and NK cell lymphomas involving the lung parenchyma, are seldom reported. Tamura and co-workers reported 24 cases of primary pulmonary lymphoma, only one of which had originated in the T-cells [13]. The PubMed database was searched going back to 1990, and only 16 cases of T-cell lymphoma were found [6]. Primary lung NK/T cell lymphoma is more rare, and only four cases have been reported in the literature [6-8].

Clinically, patients with primary lung NK/T cell lymphoma usually present with cough, fever, and dyspnoea. Treatment with antibiotics does not improve fever. Pleural effusion has also been reported. The most common radiographic findings are bilateral diffuse nodular lesions with mass-like consolidation. Histopathologically, nasal-type NK/T cell lymphoma has a characteristic histologic pattern, which is often angiocentric with prominent necrosis and vascular destruction. For this reason, most NK/T lymphomas may show extensive necrosis and are thus easily misdiagnosed as infectious lesions. Immunohistochemically, the tumor cells tend to express CD56, cytoplasmic CD3ϵ, CD2, cytotoxic granule proteins, granzyme B, and TIA-1 but not surface CD3. Of course, some special cases, such as CD20-positive NK/T-cell lymphoma, have been reported [14-16]. In this case, the tumor cells were negative for CD20. Thus, a diagnosis of NK/T cell lymphoma was first considered based on the histopathological characteristics and typical immunohistochemical features outlined above. Moreover, there were no skin eruptions, and no evidence of lymphoma involvement was found in the nasal endoscopy and positron emission tomographic (PET) imaging. A bone marrow biopsy was also negative. In this way, a diagnosis of primary pulmonary extranodal NK/T cell lymphoma, nasal type was made.

The article "Identification of genuine primary pulmonary NK cell lymphoma via clinicopathologic observation and clonality assay" was published in 2013. Journal: Diagn Pathol.

Extranodal NK/T cell lymphoma is an uncommon subtype of NHL. It is derived from either activated NK cells or, rarely, cytotoxic T-cells [17]. If a patient with NK or T-cell tumors has unusual reactions to treatment or unusual prognosis [18], it is better to differentiate the NK tumors from the T-cell tumors in our opinion. Simultaneously, several studies have demonstrated that it is necessary to elucidate the origin of NK/T cell lymphoma [18,19]. Unfortunately, related research is still very limited. Thus, our issue is to determine whether the tumor originated from NK or T cells.

Monoclonality is one of the main features of most tumors, but normal and reactive hyperplastic lesions are polyclonal [20]. Clonal analysis techniques, including T-cell and B-cell receptor gene rearrangement and one technique based on X-chromosome inactivation mosaicism and polymorphisms at the PGK and AR loci in female somatic cells, play an important role in differentiating neoplasm from reactive hyperplasia. In particular, T-cell receptor (TCR) gene rearrangement may be used to distinguish NK/T-cell lymphoma from T-cell lymphoma. If TCR gene rearrangement shows a clonal pattern, the tumor is of T-cell origin. If negative, a diagnosis of NK/T cell lymphoma can be made [21]. The point has been confirmed by many NK/T cell lymphoma reported in the literature [22]. That is to say, determination of TCR gene rearrangement by PCR-based analysis may not be useful for making diagnosis of extranodal NK/T cell lymphoma. In the present study, DNA was isolated from paraffin-embedded tissue samples and analyzed for TCR gene rearrangement using PCR-based techniques. The results showed no evidence of clonal gene rearrangement. As pointed out by Mansoor et al., this condition seemed to be diagnosed as NK-cell lymphoproliferative lesions, specifically polyclonal lesions [23]. However, the truth of the matter was quite different.

Clonality assays, which are based on X-chromosome inactivation mosaicism and polymorphisms at the PGK and AR loci in female somatic cells, are a very important means of differentiating neoplasm from reactive hyperplasia. The principle behind this assay is that each female somatic cell contains two X chromosomes, one of which is randomly inactivated by methylation during early embryogenesis and the other of which retains its genetic activity throughout life. PGK gene polymorphism shows the presence of a single nucleotide polymorphic site identified by *Bst* XI located downstream of the methylation site. AR polymorphism shows different lengths of CAG short-tandem repeats (STR) at exon 1 [24]. After digestion with the methylation-sensitive restriction enzyme *Hha* I, normal and reactive hyperplastic tissues with polymorphisms show two alleles of equal intensity. Neoplastic tissues show only one of the two alleles, with obviously reduced intensity. This lesion should be diagnosed as true NK cell lymphoma or T cell lymphoma if it shows a monoclonal pattern based on the histopathological features, immunohistochemical characteristics, and TCR. In the present study, the clonal status of the lesion was evaluated using laser microdissection and a clonal assay to further confirm the conclusion. The results demonstrated that the lesion was monoclonal hyperplasia, which supported the diagnosis of true NK-cell lymphoma. Six of the eight patients described by Mansoor et al. were female [23]. For this reason, clonality assays are here recommended as a means of confirming the nature of these lesions. Moreover, TCR gene rearrangement was not performed in any of the four cases reported in the literature [6-8]. This suggests that the diagnosis of NK cell lymphoma of the lung was not confirmed. Of course, this method has its limitations. Specifically, it can only be used to analyze samples from female individuals. Thus, the diagnosis of most patients with NK/T cell lymphoma still depends upon morphology, immunophenotype, EBER in situ hybridization, and TCR gene rearrangement.

The article "Identification of genuine primary pulmonary NK cell lymphoma via clinicopathologic observation and clonality assay" was published in 2013. Journal: Diagn Pathol.

Remarkably, there are many similarities between extranodal NK/T cell lymphoma with advanced stage and aggressive natural killer cell leukemia/lymphoma, such as the morphology, immunophenotype, germline configuration of TCR gene and EBV association [25]. However, Kwong et al. [26] has pointed out the latter can be different from the former by the absence of a previous history, a shorter illness, a younger age of presentation and an extremely aggressive course. In our case, the blood count was normal, and the tumor cells did not involve in bone marrow, liver, and spleen. Moreover, the patient was an older female except showing a short survival time. Thus, we considered that it should be diagnosed as extranodal NK/T cell lymphoma.

The prognosis of primary pulmonary NK/T-cell lymphoma is very poor, although aggressive treatments with CHOP-based chemotherapy and surgical resection have been reported in the literature. Among the four patients with primary pulmonary NK/T cell lymphoma, the longest life expectancy was less than 6 months [5]. Recently, some studies demonstrated that the expression of both LMP1 and LMP2A showed significant correlations with the prognosis of patients with extranodal NK/T cell lymphoma [27]. In our case, the tumor cells were positive for LMP1. Therefore, the patient died 1 month after leaving the hospital, which supported the conclusion. Moreover, it appears to be very difficult to diagnose NK/T cell lymphoma because of the associated extensive necrosis and variable morphology. In the present case, frozen sections were examined twice during the operation, and the results showed microscopically extensive coagulative necrosis. Fortunately, the patient underwent a lobectomy and consented to allow pathologists to examine a large number of sections.

The article "Identification of genuine primary pulmonary NK cell lymphoma via clinicopathologic observation and clonality assay" was published in 2013. Journal: Diagn Pathol.

In conclusion, this is the first reported case of genuine primary pulmonary NK cell lymphoma. Pathologists should carefully investigate the whole lesion when extensive coagulative necrosis with atypical lymphocyte infiltration is observed in a major lesion. This renders primary pulmonary NK cell lymphoma less likely to be misdiagnosed as an infectious lesion. In addition, TCR gene rearrangement and clonal assays based on the polymorphisms of PGK and AR and X-chromosomal inactivation mosaicism should be performed in any somatic tissue samples taken from female patients.

## Competing interests

The authors declare that they have no competing interests.

## Authors’ contributions

LG selected the research topic, participated in the study, and wrote the manuscript. LXW provided the CT image. GSH performed the diagnosis, and wrote the manuscript. LW carried out TCR gene rearrangement. WDZ participated in writing the manuscript. YHL and WZ provided grant support. SJZ, LY, and XJH conducted the pathological examination. ML provided the technique support. All authors have read and approved the final manuscript.
